# A Comparison among Different Machine Learning Pretest Approaches to Predict Stress-Induced Ischemia at PET/CT Myocardial Perfusion Imaging

**DOI:** 10.1155/2021/3551756

**Published:** 2021-11-27

**Authors:** Rosario Megna, Mario Petretta, Roberta Assante, Emilia Zampella, Carmela Nappi, Valeria Gaudieri, Teresa Mannarino, Adriana D'Antonio, Roberta Green, Valeria Cantoni, Parthiban Arumugam, Wanda Acampa, Alberto Cuocolo

**Affiliations:** ^1^Institute of Biostructure and Bioimaging, National Council of Research, Naples, Italy; ^2^IRCCS-SDN, Naples, Italy; ^3^Department of Advanced Biomedical Sciences, University Federico II, Naples, Italy; ^4^Department of Nuclear Medicine, Central Manchester Foundation Trust, Manchester, UK

## Abstract

Traditional approach for predicting coronary artery disease (CAD) is based on demographic data, symptoms such as chest pain and dyspnea, and comorbidity related to cardiovascular diseases. Usually, these variables are analyzed by logistic regression to quantifying their relationship with the outcome; nevertheless, their predictive value is limited. In the present study, we aimed to investigate the value of different machine learning (ML) techniques for the evaluation of suspected CAD; having as gold standard, the presence of stress-induced ischemia by ^82^Rb positron emission tomography/computed tomography (PET/CT) myocardial perfusion imaging (MPI) ML was chosen on their clinical use and on the fact that they are representative of different classes of algorithms, such as deterministic (Support vector machine and Naïve Bayes), adaptive (ADA and AdaBoost), and decision tree (Random Forest, rpart, and XGBoost). The study population included 2503 consecutive patients, who underwent MPI for suspected CAD. To testing ML performances, data were split randomly into two parts: training/test (80%) and validation (20%). For training/test, we applied a 5-fold cross-validation, repeated 2 times. With this subset, we performed the tuning of free parameters for each algorithm. For all metrics, the best performance in training/test was observed for AdaBoost. The Naïve Bayes ML resulted to be more efficient in validation approach. The logistic and rpart algorithms showed similar metric values for the training/test and validation approaches. These results are encouraging and indicate that the ML algorithms can improve the evaluation of pretest probability of stress-induced myocardial ischemia.

## 1. Introduction

Artificial intelligence has assumed a consolidated role in numerous fields and also in the healthcare and research and development. Machine learning (ML), an application of artificial intelligence that refers to computational algorithms designed to learn from experience, has been used successfully for diagnosis, prognosis, and drug development [1–4]. Among the recommendations for ML implementation in clinical research, there is data normalization, feature selection, parameter tuning, and independent validation [5, 6].

In the field of cardiology, the search for methods for obtaining reliable pretests probability of disease has been underway for some time [7]. These tools should assist the physician in making decisions about referring patients for examination. Usually, for the prediction of coronary artery disease (CAD), traditional risk factors, such as age, gender, chest pain, and comorbidity related to cardiovascular diseases, such as hypertension, diabetes, and hyperlipidemia, are considered. These variables are analyzed by logistic regression to quantifying their relationship with the outcome of the exam and obtaining predictions for new patients [8–11]. However, the models obtained by these studies do not show a great performance, probably due to the declining prevalence of CAD and because the evaluation for CAD has shifted to older patients, more women, and more patients with atypical symptoms than in previous decades [12]. Including in the model, other clinical, laboratory, and instrumental characteristics could improve prediction accuracy; however, adding variables may be expensive and time-consuming and also incorrectly reclassify patients with suspected CAD. Using publicly available dataset, it has been recently reported that ML algorithms have high accuracy to detect the presence of CAD [13]. Yet, if the application of more complex algorithms on traditional risk factor may optimize the estimation of pretest probability of CAD, it remains to be defined. In the present study, we aimed to investigate the potential of different ML techniques for the evaluation of suspected CAD, having as gold standard the presence of stress-induced ischemia by ^82^Rb positron emission tomography/computed tomography (PET/CT) myocardial perfusion imaging (MPI).

In summary, the main contributions of this work include the following:

1. A comparison of the value of several ML algorithms in predicting the presence of stress-induced ischemia by noninvasive cardiac imaging
2. We selected ML algorithms based on their use in the medical field and on the fact that they are representative of different classes of algorithms, such as deterministic, adaptive, and decision tree

The rest of this paper is organized as follows.  Section 2 describes the method with detailed information of datasets and ML techniques used.  Section 3 describes the results. The discussion is presented in Section 4 followed by the conclusions in Section 5.

## 2. Materials and Methods

### 2.1. Study Design and Eligibility

Our cohort included a total of 2503 consecutive patients, who underwent cardiac ^82^Rb PET/CT for suspected CAD as part of their diagnostic program between June 2010 and October 2019. Patients with known CAD and patients with acute coronary syndrome were excluded. A patient was considered to have known CAD at the time of imaging based on a provided history of previously diagnosed atherosclerotic coronary disease, history of myocardial infarction (chest pain or equivalent symptom complex, positive cardiac biomarkers, or typical electrocardiographic changes), history of percutaneous coronary intervention, or history of coronary artery bypass grafting. For patients undergoing more than one PET/CT study, only the earliest procedure was considered. All patients were part of ongoing prospective dedicated database [14]. This study complies with the Declaration of Helsinki. The review committee of our institution approved this study (Ethics Committee, University Federico II, protocol number 110/17), and all patients gave informed consent.

### 2.2. Clinical Definitions

Chest pain was classified according to the American College of Cardiology/American Heart Association 2002 guideline update on exercise testing [15]. Patients were considered as having diabetes if they were receiving treatment with oral hypoglycemic drugs or insulin. A family history of premature CAD was defined as a diagnosis of CAD in a first-degree relative prior to or at 55 years of age. Hypertension was defined as a blood pressure > 140/90 mm Hg or use of antihypertensive medication. Hyperlipidemia was defined as total cholesterol level > 6.2 mmol/L or treatment with cholesterol lowering medication. Smoking history was defined as prior or current tobacco use. Body mass index (BMI) was dichotomized with cut-off to 30, according to obesity definition.

### 2.3. PET/CT Imaging

As a routine preparation for ^82^Rb cardiac PET/CT, patients were asked to discontinue taking methylxanthine containing foods or beverages for 24 hours. Scans were acquired using a Biograph mCT 64-slice scanner (Siemens Healthcare). Rest and stress cardiac PET/CT images were acquired as follows: scout CT was performed to check patient position, and low-dose CT (0.4 mSv; 120 kVp; effective tube current, 26 mA [11-mAs quality reference]; 3.3 seconds) was performed for attenuation correction, during normal breathing before and after PET acquisitions. For both rest and stress images, 1110 MBq of ^82^Rb was injected intravenously with a 7-minute list-mode PET acquisition. Dynamic PET acquisition was started at rest followed by adenosine pharmacologic stress (140 *μ*g × kg^−1^ × min^−1^ for 4.5 minutes, with tracer administration between 2 and 2.5 minutes). Rest and stress dynamic images were reconstructed into 26-time frames (12 × 5 seconds, 6 × 10 seconds, 4 × 20 seconds, and 4 × 40 seconds; total, 6 minutes) using the vendor standard ordered subsets expectation maximization 3D reconstruction (2 iterations, 24 subsets) with 6.5 mm Gaussian postprocessing filter. In addition, the images were corrected for attenuation using the low-dose CT. The heart rate, systemic blood pressure, and 12-lead ECG were recorded at baseline and throughout the infusion of adenosine. An automated software program (e-soft, 2.5, QGS/QPS, Cedars-Sinai Medical Center, Los Angeles, CA) was used to calculate the scores (summed stress score, summed rest score, and summed difference score) incorporating both the extent and severity of perfusion defects, using the standardized segmentation of 17 myocardial regions [16, 17]. A summed difference score ≥ 2 was considered ischemic.

### 2.4. Statistical Analysis

Statistical analysis was performed using the *R* software, version 3.6.2 (The *R* Foundation for Statistical Software, Vienna, Austria). Two-sided *P* values <0.05 were considered statistically significant. The dataset consisted of 11 features, of which 10 demographic or clinical variables (age, gender, BMI, typical or atypical chest pain, diabetes mellitus, dyspnea, family history, hypertension, hyperlipidemia, smoking), and the diagnostic question with two categories: diagnostic or presurgery evaluation. Age and BMI continuous variables were categorized (<55, 55-65, >65 years, and BMI < 30); then, all data were expressed as percentages. Differences between groups were analyzed by *χ*^2^ test. The correlation among features was tested by Spearman *ρ* coefficient, embedded in the corrplot package. This nonparametric test is appropriate to evaluate the correlation between categorical variables and to find redundant features. Data in input to ML algorithms were normalized. Sensitivity, specificity, and accuracy were computed using the *c*onfusionMatrix function embedded in the caret package. Sensitivity evaluated how good a ML is for detecting the positive patients (i.e., ischemic according to MPI results), and its numeric value was obtained by ratio between the number of patients correctly assessed as positive by ML and the number of positive patients. Specificity evaluated the negative patients (i.e., normal according to the MPI results), and it was calculated by ratio between the number of patients correctly assessed as negative by ML and the number of negative patients. Accuracy measured how correctly a ML identified and excluded a given condition, and it was obtained from the ratio between the number of patients correctly assessed by ML and the total number of patients. Receiver operating characteristic curve is a graphic presentation of the relationship between sensitivity and specificity, whereas the area under this curve provides a measurement of the correct evaluation of ML with respect a random classifier. The areas under the receiver operating characteristic (AUROC) curves were computed by the *pROC* package.

### 2.5. ML Techniques

For the comparison presented in this study, we selected supervised ML algorithms, appropriate to categorical data for a binary response. We used the algorithms developed in *R*. ADA is a classification tree based on adaptive algorithms, used to fit a variety stochastic boosting. This algorithm can be used in conjunction with other types of learning procedures to improve performance. The output of these procedures, called weak learners, is combined into a weighted sum that represents the final output of the boosted classifier [18]. AdaBoost is a classifier similar to ADA, differing from this for the AdaBoost.M1 algorithm implemented by Freund and Schapire [19]. Logistic algorithm used in this study is a part of generalized linear models [20]. This classifier was chosen as a reference because adopted in clinical statistical analysis, with categorical or numerical data and dichotomous response. The equation assumed a linear relationship between the predictor variables *x*_*i*_ and the log odds (in term of probability *p*) of the event, as follows:

(1) $$\begin{array}{c} \log\frac{p}{1-p}=\beta_{0}+\overset{n}{\underset{i=1}{\sum }}\beta_{i}x_{i}. \end{array}$$

Then, the *β* coefficients are determinates, with *β*_0_ representing the particular case with all variables equal to zero. The Naïve Bayes is a probabilistic classifier based on the Bayes' theorem. This algorithm requires a strong (naïve) independence assumption between the features [21]. Random Forest is an algorithm based on an ensemble learning method for classification and regression that operate by constructing a multitude of decision trees at training time. The procedure returns as output the class that is the mode of the classes (for classification) or average prediction (for regression) of the individual trees [22]. Rpart is a decision tree algorithm that works by splitting in two parts the dataset recursively. For each step, the split is obtained considering the feature that results in the largest possible reduction in heterogeneity of the outcome variable [23]. Support vector machine (SVM) is an algorithm that constructs hyperplanes in a high-dimensional space, which can be used for classification and regression [24]. SVM is a robust prediction method that can efficiently perform nonlinear classifications, by appropriate kernels. XGBoost is a scalable end-to-end tree boosting method, based on a sparsity-aware algorithm for sparse data and weighted quantile sketch for approximate tree learning [25].

### 2.6. Approaches Used for the ML Evaluation

To testing the ML performances, the data were split randomly into two parts: training/test (80%) and validation (20%). For the training/test of data, we applied a 5-fold cross-validation method, repeated 2 times. With this subset, we performed the tuning of free parameters for each algorithm. For both training/test and validation, we computed accuracy, sensitivity, specificity, and AUROC.

### 2.7. Hardware and Software Characteristics

For this study, we used a common personal computer equipped with a 2.2 GHz Intel i3-2330 quad-core processor, 8 GB of RAM, and a 0.5 TB SSD. The operating system was a Windows 10, whereas the scripts in *R* programming code were obtained developing inhouse software.

## 3. Results

Demographic and clinical characteristics of study population according to normal or ischemic MPI response are summarized in Table 1. All features, except BMI and smoking, were statistically significant to *χ*^2^ test.

Figure 1 shows the Spearman correlation coefficients matrix of features. All the found absolute values were <0.25, highlighting only weak correlations among features. The cluster with higher correlation among features was obtained by diabetes, hypertension, and hyperlipidemia (*ρ* = 0.22). The very low correlation values demonstrated the absence of redundant features.

Figure 2 reports the feature importance for each algorithm. We observed the same feature importance values for ADA and AdaBoost algorithms, whereas small differences (<5%) were found between these procedures and the Naïve Bayes ML. Therefore, we reported a unique bar plot for these three algorithms. In general, the most important features were age and gender, followed from diabetes or chest pain. We also observed relevant differences among features importance of most of ML algorithms, except for the two adaptive and Naïve Bayesian algorithms. In fact, for these three algorithms, the importance values were comprised between 0.50 and 0.65, whereas for the logistic algorithm, we obtained larger interval of values from 0.001 to 0.93.

Table 2 summarizes the space parameters and the value chosen for the tuning of ML. Parameters were tested using a 5-fold cross-validation, repeated 2 times, targeted to maximize the C-index. Among all tested setting for each algorithm, we chose the combination with higher sensitivity to balance the result performances.

Table 3 shows the C-statistics results of the ML algorithms, for training/test and validation approaches. In general, the performances in training/test approach were better than of the validation approach. Due to unbalanced dataset, specificity resulted greater than sensitivity. For all metrics, the best performance in training/test was observed for AdaBoost ML. The Naïve Bayes ML resulted to be more efficient in validation approach. ML based on traditional logistic algorithm showed a low sensitivity and similar performance for the training/test and validation approaches.  Figure 3 shows a graphical comparison among the ROC curves of the ML algorithms, for both training/test and validation approaches.

Figure 4 shows the tree generated from the rpart algorithm. To make the decision tree easier to read, the max depth was fixed to 5. The first spit was on age and for younger patients (≤65 years), without any node until the terminal leaf, where a prevalence of normal MPI of 86% was observed. For older patients (>65 years), the algorithm calculated the gender node, with a percentage of normal MPI of 70%. The split in this node, related to the female gender, was followed by diabetes, chest pain, and family history of CAD.

## 4. Discussion

At best of our knowledge, this is the first study comparing the value of several ML algorithms in predicting the presence of stress-induced ischemia by ^82^Rb PET/CT cardiac imaging. We selected eight ML algorithms based on their clinical use and on the fact that they are representative of different classes of algorithms, such as deterministic (e.g., SVM), adaptive (e.g., ADA), and decision tree (e.g., rpart). The results indicate that by adaptive (ADA and AdaBoost) and Random Forest algorithms, AUROC curve was ≥90% in training/test phase.

As input features for the ML algorithms, we considered demographic data and traditional cardiac risk factors. No significant correlations were detectable between variables, a necessary condition for features selection in ML techniques and for data processing. The feature importance is an important step for ML techniques. In our study aside from demographic characteristics, diabetes and chest pain resulted to be the most useful features for predicting stress-induced ischemia by PET/CT. This result confirms another study based on SPECT, where the feature importance, obtained by logistic regression, was the following: gender, age, and chest pain [26]. Noteworthy, features (*BMI* and smoking) showing not significant *χ*^2^ statistic resulted relevant at ML analysis. Indeed, ML algorithms may capture the subtle value of features apparently not significant at conventional analysis.

The ML algorithms showed a variable accuracy (72%-89%) by training/test phase, with low sensitivity and high specificity. This latter finding probably reflects the unbalanced dataset between normal and abnormal MPI and is in agreement with the observation that, in the contemporary pretest probability of CAD, noninvasive imaging tests have greater ruling out that ruling in capabilities [12]. Also, the AUROC values were very wide (61%-95%), with better performances for ADA, AdaBoost, and Random Forest. By these ML algorithms, we obtained the greater values of sensitivity. However, these better performances were lower in the validation set, probably due to the ensemble of weakly solutions and a high number of decision trees elaborated during the training/test phase for each of the three ML algorithms. For XGBoost, we observed a similar performance to these three algorithms, but a lower sensitivity. The Naïve Bayes and SVM resulted to have more generalized performances by the two approaches, with lightly better results by validation phase. The logistic and rpart algorithms showed similar metric values for the training/test and validation approaches.

The logistic technique, taken as a reference, did not result particularly performant with respect to the other ML algorithms. In particular, the value of sensitivity was the lowest, probably explainable with the unbalanced dataset. However, the AUROC resulted higher with respect to a similar study (AUROC = 64%) based on clinical risk factors, single-photon emission computed tomography imaging, and logistic regression [10].

As an example of a tool for decision-making, we reported the tree obtained by rpart. From a graphic point of view, it is immediate to verify the effect of age and *gender* on the construction of the decision tree. For younger patients, there is a prevalence of normal MPI, without further ramifications. Otherwise, a gender split is observed, followed in both cases by the split of diabetes and chest pain, with a larger complexity for the male gender.

Previous studies used ML algorithms in cardiology [27], but at the best of our knowledge, no study evaluated this approach to estimate the pretest probability of an ischemic response to PET/CT. In a study based, an XGBoost ML was developed in a large series of symptomatic patients to predict pretest probability of obstructive CAD on coronary computed tomography angiography. The ML model had significantly higher discrimination (AUROC = 81%), as compared to traditional models, with a good sensitivity (91.9%) but a low (38.8%) specificity. This study was used a 10-fold cross-validation approach but and no independent validation dataset [28]. In another study [29], a SVM algorithm was used to determine the diagnostic value of joint PET myocardial perfusion and metabolic imaging for predicting obstructive coronary artery disease in symptomatic patients with available coronary angiography. The study included only 88 patients, most of them with known CAD. The joint PET evaluation improves had a good performance (AUROC = 86%), and the SVM algorithm outperformed the other methods evaluated. In a study [30], including a total of 16,120 patients, ML improved one-year risk discrimination in predicting durable left ventricular assist devices as compared to logistic regression (C-index 71% vs. 69%, *P*  < 0.001); however, calibration metrics were comparable. Globally, these studies confirm limited value of current clinical models to accurately predict the presence of myocardial ischemia at stress MPI [31].

## 5. Conclusions

The results of this study performed in a large series of patients with suspected CAD demonstrate that the classification based on demographic and cardiovascular risk factors has a limited value in validation phase for predicting an ischemic response by ^82^Rb PET/CT in patients with suspected CAD. We selected eight ML algorithms that are implemented by different software packages and can be used by other researchers on their MPI data. Other ML algorithms, such as monarch butterfly optimization [32], earthworm optimization algorithm [33], elephant farming optimization [34, 35], moth search algorithm [36], slime mould algorithm [37], and Harris hawks optimization [38], can also be used to predict stress-induced ischemia by MPI and should be tested in future studies. In conclusion, the role of other clinical and instrumental characteristics, as well as developing and perfecting more complex algorithms to improve the prediction of stress-induced ischemia by MPI, remains a work in progress.

## Figures and Tables

**Figure 1:** Correlation matrix of the features used. The matrix elements are displayed in hierarchical clustering order. The numbers indicate the Spearman *ρ* coefficient between two features.

**Figure 2:** Importance of the features for each ML algorithm. ADA, AdaBoost, and Naïve Bayesian features importance were grouped into a single bar plot as the values for the two adaptive algorithms turned out to be equals, and Naïve Bayesian values differed with them by less than 5%.

**Figure 3:** Comparison among the ROC curves of the eight ML techniques considered. The ML performances are reported separately for the training/test approach (a) and validation approach (b). Parenthesis are reported the AUROC values.

**Figure 4:** Decision tree obtained by rpart algorithm. Each node or leaf is reported the prevalence concerning MPI outcome (nor: normal; isch: ischemic), the ratio between the number of prevalent and total patients, and the relative percentage.

**Table 1:** Clinical characteristics of cohort according to MPI outcome.

	Normal (*n* = 2002)	Ischemic (*n* = 501)	*P* value
Age, *n* (%)			<0.001
<55	777 (39)	84 (17)	
55-65	603 (30)	146 (29)	
>65	622 (31)	271 (54)	
Male gender, *n* (%)	881 (44)	334 (67)	<0.001
Body mass index ≥30, *n* (%)	1024 (51)	258 (52)	0.93
Chest pain, *n* (%)			<0.001
Typical	678 (34)	114 (23)	
Atypical	256 (13)	87 (17)	
Noncardiac^∗^	1068 (53)	300 (60)	
Diabetes, *n* (%)	479 (24)	187 (37)	<0.001
Dyspnea, *n* (%)	446 (22)	139 (28)	<0.05
Family history of CAD, *n* (%)	945 (47)	199 (40)	<0.005
Hypertension, *n* (%)	1361 (68)	401 (80)	<0.005
Hyperlipidemia, *n* (%)	1210 (60)	343 (69)	<0.005
Smoking, *n* (%)	557 (28)	144 (29)	0.72
Diagnostic question, *n* (%)^§^			<0.001
Diagnostic evaluation	1642 (82)	370 (74)	
Presurgery evaluation	360 (18)	131 (26)	

^∗^Considering noncardiac patients as the reference. ^§^Considering diagnostic evaluation patients as the reference.

**Table 2:** Values used for tuning of parameters for each ML technique.

	Parameter	Parameter space	Chosen value
ADA	Number of trees	10, 25, 50, 100, 200	25
	Max tree depth	5, 10, 20, 50	10
	Learning rate	0.001, 0.005, 0.01, 0.05, 0.1, 0.5	0.01

AdaBoost	Number of trees	10, 25, 50, 100, 200	50
	Method	AdaBoost.M1, real AdaBoost	AdaBoost.M1

Logistic	Family	Binomial	Binomial

Naïve Bayes	Laplace correction	0, 0.5, 1.0	0
	Distribution type (kernel)	True, false	False
	Bandwidth adjustment	0.01, 0.05, 0.1, 0.5, 1.0	0.1

Random Forest	Number of randomly selected predictors	3, 5, 10, 20	10

Rpart	Minimum number of observations in a node	10, 15, 30	15
	Minimum number of observations in any leaf node	3, 5, 10	5
	Max tree depth	3, 5, 10, 20	10
	Complexity parameter of the tree	0.0001, 0.001, 0.01, 0.1	0.001

SVM	Kernel	Linear, radial, sigmoid	Sigmoid
	Parameter needed for sigmoid	0.05, 0.1, 0.25, 0.5	0.1
	Cost	0.5, 1, 2, 5	1

XGBoost	Number of trees	25, 50, 100, 200	100
	Max tree depth	5, 10, 20	10
	Learning rate	0.001, 0.005, 0.01, 0.05, 0.1, 0.5	0.01
	Subsamples	0.5, 0.75, 1	1

**Table 3:** Metrics obtained from the ML techniques, evaluated on training/test and validation approaches.

	Training/test (*n* = 2003)				Validation (*n* = 500)			
	Accuracy (%)	Sensitivity (%)	Specificity (%)	AUROC (%)	Accuracy (%)	Sensitivity (%)	Specificity (%)	AUROC (%)
ADA	88	48	97	90	76	26	89	68
AdaBoost	89	67	95	95	71	23	87	66
Logistic	80	5	98	72	80	7	98	75
Naïve Bayes	77	23	91	70	80	27	92	73
Random Forest	89	51	98	93	75	21	89	65
Rpart	82	27	96	75	76	17	91	70
SVM	72	13	87	61	77	21	91	65
XGBoost	83	27	97	83	77	18	92	69

## Data Availability

The data used in this study are available from the corresponding author on a reasonable request.
